The article "Effects of ADOPT-Based Breathing Training Combined with Continuous Nursing on Quality of Life, Mental Health, and Self-Efficacy in Lung Cancer Patients Undergoing Chemotherapy: Based on a Retrospective Cohort Study" was retracted in 2023. Reasons: unreliable results or conclusions; lack of ethics approval or compliance; concerns about the data; concerns about the results or conclusions.

# Effects of ADOPT-Based Breathing Training Combined with Continuous Nursing on Quality of Life, Mental Health, and Self-Efficacy in Lung Cancer Patients Undergoing Chemotherapy: Based on a Retrospective Cohort Study

**DOI:** 10.1155/2022/4164771

**Published:** 2022-04-20

**Authors:** Ji Mou, Senzhong Zheng

**Affiliations:** Department of Pulmonary and Critical Care Medicine, Taizhou First People's Hospital, Taizhou 318020, China

## Abstract

**Objective:**

Considering the poor effect of routine nursing program on patients with lung cancer after chemotherapy, a retrospective cohort study was conducted to elucidate the effects of respiratory training based on ADOPT mode combined with continuous nursing on quality of life, mental health, and self-efficacy in patients undergoing lung cancer chemotherapy.

**Methods:**

Sixty patients with lung cancer admitted in our hospital from January 2019 to April 2021 were selected. Patients in both groups received ADOPT breathing training. Patients who underwent routine nursing were assigned into control group (*n* = 30) and patients with continuous nursing were set as study group (*n* = 30). The differences in nursing satisfaction, self-management efficacy, quality of life score, mental health, family care index, and self-transcendence scale scores of patients with lung cancer were determined.

**Results:**

First of all, we compared the baseline data of the two groups, and there was no statistical difference. In the comparison of nursing satisfaction between the two groups, 24 cases in the study group were very satisfied, 5 cases were satisfied, 1 case was general, and the satisfaction rate was 100%, whereas in the control, 14 cases were very satisfied, 8 cases were satisfied, 4 cases were not satisfied, and the satisfaction rate was 86.67%. Compared to the control, the nursing satisfaction was higher in the study group (*P* < 0.05). There exhibited no significant difference in the sense of self-management efficacy between the two on the day of admission (*P* > 0.05). After nursing, the scores of self-management efficacy were higher in the study group, compared to the control (*P* < 0.05). In contrast to control, the scores of self-management efficacy at discharge and 1, 3, and 6 months after discharge were higher in the study group (*P* < 0.05). In terms of the scores of quality of life of patients with lung cancer, on the day of admission, no significant difference exited (*P* > 0.05). The scores of quality of life at discharge and 1, 3, and 6 months after discharge of the study group were higher compared to the control (*P* < 0.05). In the comparison of mental health, there was no significant difference between the two groups on the day of admission (*P* > 0.05), but the scores of anxiety and depression in the two groups decreased after nursing, and the scores of anxiety and depression in the study group at discharge and 1 month, 3 months, and 6 months after discharge were lower than those in the control group (*P* < 0.05). In terms of the family care index, there was no significant difference between the two groups at admission (*P* > 0.05), but after nursing, the family care index of the two groups increased, and the family care index at discharge and 1, 3, and 6 months after discharge was greater in the study group (*P* < 0.05). In terms of the score of self-transcendence scale, there exhibited no significant difference on the day of admission (*P* > 0.05), but the score of self-transcendence scale of the two groups increased after nursing. Furthermore, compared to the control, the score of self-transcendence scale at discharge and 1 month, 3 months, and 6 months after discharge in the study group was higher (*P* < 0.05).

**Conclusion:**

Patients undergoing lung cancer chemotherapy using ADOPT-based breathing training combined with continuous nursing can effectively facilitate the overall quality of life of lung cancer chemotherapy patients, promote the mental health and self-efficacy of patients with lung cancer chemotherapy, and then reduce the medical burden of patients. The nursing model based on ADOPT breathing training combined with continuous nursing is worthy to be applied in the rehabilitation of patients with lung cancer.

## 1. Introduction

Lung cancer remains one of the most common malignant tumors with high mortality all over the world. Survival analysis demonstrated that lung cancer patients had a short survival time, with a 1-year survival rate of 42% and a 5-year survival rate of only 16% [1]. At present, the early diagnosis of lung cancer is very difficult. Until now, 70%-80% of the patients are diagnosed within the advanced stage, losing the opportunity for surgery, and most of them are treated mainly by chemotherapy [2]. The most common side effects of chemotherapy patients are myelosuppression, liver and kidney injury, gastrointestinal tract, pulmonary toxicity, and so on. In severe cases, it will affect the progress of chemotherapy and even endanger the lives of patients. Therefore, patients with advanced lung cancer suffer great physical and mental pain; face adverse reactions caused by chemotherapy, fear of death, weakening of role function, etc.; and reduce their quality of life [2]. On the other hand, many toxic and side effects of chemotherapy patients do not necessarily occur during hospitalization, and there is a lag. A variety of studies have confirmed that lung cancer patients after discharge have greater information and nursing needs [2]. Therefore, patients should be provided with high-quality and efficient holistic care to improve their quality of life after returning home. ADOPT model is a problem-solving model put forward by American scholars in 2006, which consists of five steps: A (Attitude): individual attitude and expectation; D (Definition): individual identification of current obstacles and objective understanding of the nature of the problem; O (open mind): individual thinking about new and creative ways to solve problems; P (Planning): individual determines feasible strategies; and T (Try it out/Experiment): individuals implement the strategy and evaluate the results, adjust the strategy if necessary, and start a new plan [3]. Therefore, in this study, ADOPT model was incorporated into the respiratory training of patients undergoing lung cancer surgery, in order to solve the problems encountered by patients in respiratory training in time, make patients actively participate in respiratory training, and promote their rehabilitation.

Continuous nursing is developed on the basis of holistic nursing theory, in order to meet the actual needs of discharged patients under different health service systems or different conditions of the same health service system and to provide patients with an orderly, coordinated, and continuous care behavior [4]. The continuous nursing model has been relatively mature, and it has been proved that it can provide better extended care for patients, and remarkable results have been achieved, which mainly includes guided nursing model, geriatric resource model, continuous nursing intervention model, and APN (senior practice nurse) continuous nursing model. Some studies have shown that the continuous nursing model has strong practicability in reducing the number of hospitalization of patients, reducing the rate of reconsultation, reducing medical expenditure, and improving their quality of life. The research on continuous nursing in China started relatively late, and there is no perfect continuous nursing model. At present, continuous nursing in China mainly adopts the way of telephone follow-up. There are few reports on continuous nursing of lung cancer patients undergoing chemotherapy, and there are few randomized controlled studies on the use of continuous nursing. However, there are few reports on the combination of respiratory training based on ADOPT mode and continuous nursing. Therefore, a retrospective cohort study was conducted to survey the influence of respiratory training based on ADOPT mode combined with continuous nursing on life quality, mental health, and self-efficacy of lung cancer patients undergoing chemotherapy.

## 2. Cases and Methods

### 2.1. General Patient Information

Sixty lung cancer patients admitted in our hospital from January 2019 to April 2021 were selected. Patients in both groups received ADOPT breathing training. Patients who underwent routine care were assigned into control group (*n* = 30), and patients with continuous care were set as study group (*n* = 30). In the control group, the age was 43-74 years old, with 65.67 ± 3.57 average years, including 18 males and 12 females; education: 11 cases with junior high school or below education, 12 cases with high school education, and 7 cases above senior high school; pathological types: 3 cases of small cell lung cancer and 27 cases of non-small cell lung cancer; and concomitant diseases: hypertension (*n* = 8), diabetes (*n* = 10), and hyperlipidemia (*n* = 12). In the study group, the age was 44-76 years old, with 65.61 ± 3.58 average years, including 16 males and 14 females; educational background: 11 cases in education of junior high school, 10 cases with education of senior high school, and 9 cases with senior high school education; pathological types: 4 cases of small cell lung cancer and 26 cases of non-small cell lung cancer; and concomitant diseases: hypertension in 7 cases, diabetes in 11 cases, and hyperlipidemia in 12 cases. There remains no statistical significance in terms of general data. This study was endorsed by the Medical Ethics Association of our hospital, with all patients signing the informed consent.

The inclusion criteria include [5] as follows: (1) patient with lung cancer were diagnosed for the first time and staged by TNM. (2) The estimated survival time is more than 3 months. (3) The age range is 18-80 years old, the cognition is normal, and can read and write words normally. (4) Know the condition and volunteer to participate in current study.

Exclusion criteria include as follows: (1) patient with unconsciousness and mental disorders, (2) those who are undergoing synchronous radiotherapy, and (3) those complicated with severe cardio-cerebrovascular diseases.

### 2.2. Treatment Method

ADOPT mode breathing training includes the following: A (Attitude): each time, the researchers evaluated patients' knowledge and attitude towards yoga breathing training and guided patients to establish a positive attitude towards yoga breathing training. In addition, the researchers believe that patients can solve the problems encountered in yoga breathing training by using some methods, so that patients have a positive attitude to face difficulties and improve their self-efficacy. D (Definition): effective problem solving is based on correct information. Patients should look at their problems objectively, understand the nature of the problems, and know what actions need to be taken to solve them. On the day of admission, the researchers introduced the purpose, method, and mechanism of yoga breathing training to patients, and issued a self-developed manual to patients. During the patient's stay in hospital, each time the researchers supervise the patient's yoga breathing training, they will work with the patient to evaluate and define the patient's current problems related to breathing training, which may make it difficult to persist in breathing training. O (Open mind): researchers encourage patients to use open and creative thinking to find ways to solve the problems or obstacles encountered in yoga breathing training, so as to improve their training compliance. Each time a patient is in hospital, the researchers encourage patients to think freely about ways to overcome the current problems defined in the previous stage each time they supervise the patient's yoga breathing training and proactively discuss their own ideas or suggestions on the problem-solving process with the researchers. P (Planning): patients review the ideas generated in the previous stage and choose feasible ways to overcome the current problems, such as family members participating in escort training and multimedia video support, and work with researchers to develop a yoga breathing training plan for each time. T (Try it out): patients perform yoga breathing training according to the plan made in the previous stage and summarize with the researchers after each breathing training to review which methods are effective and ineffective in solving current problems and enabling them to persist in breathing training. For effective methods, record and summarize in time and build up patients' confidence; for ineffective methods, analyze the reasons with patients and make new plans together.

The control group received routine nursing intervention in the department and issued the disease guidance manual to the patients on the day of admission, evaluated the admission, patiently conducted health education on patients, and explained to the patients the matters needing attention in disease-related self-management. Individualized nursing guidance is given, and the way of education is mainly through health education.

The study group carried out continuous nursing based on the control, and the specific measures were as follows:

1. To set up a continuous nursing team: the members of the team include the researcher himself, 4 responsible nurses with good professional knowledge and skills, 2 oncology nurses, 1 director of nursing department, and 1 chief physician of chemotherapy department. The director of the nursing department and the chief physician of the chemotherapy department served as research consultants and quality control, oncology nurses assisted in the formulation of continuous nursing plans, and the researchers and 4 responsible nurses were responsible for the implementation of continuous nursing care and related records of discharged patients. Before the beginning of the study, the team members were trained, including the theory, content, and intervention ways of continuous nursing and the distribution and filling of the adjustment form, and worked out the intervention plan together
2. Instruct patients to use the network platform correctly: join all patients in the WeChat group while they are in hospital, and teach older patients with low education level to learn how to use WeChat. Ensure that all patients can use WeChat correctly when they are discharged from the hospital and encourage patients' families to join and participate in the group discussion and study. On the day of discharge, the health guidance assessed the symptoms and needs of the patients, filled in the discharge schedule, and gave health education to the patients. The contents include self-monitoring of disease changes, medication knowledge, side effects of chemotherapeutic drugs and coping measures, daily activities and diet, and regular reexamination of hemogram. Let patients understand the importance of insisting on treatment and rehabilitation through health guidance. Online guidance encourages patients and their families to speak freely in WeChat groups. The researchers and four responsible nurses replied and answered questions online in a timely manner and sent relevant materials on WeChat in different periods: (1) health lecture hall of our hospital, (2) methods and pictures of catheter maintenance, (3) guidance on supplementary nutrition, (4) knowledge of diseases, (5) articles on sharing the successful experiences of anticancer patients, (6) questions and answers, (7) guidance on family care, and (8) pay attention to remind regular review of hemogram, catheter maintenance, and regular next chemotherapy. For patients with more problems and heavy burden, chat on WeChat alone to communicate with them and their families, evaluate the problems and adjust the plan in time, give relevant methods and suggestions, and encourage family members to accompany and comfort patients. The dissemination of content related to the privacy of patients is prohibited. The telephone return visit department has a special return call, which is completed by the researcher himself and the responsible nurse in the team
3. The contents of the telephone return visit include within 24 hours after the discharge of the first chemotherapy, mainly to evaluate the improvement of the existing nursing problems of the patients, to evaluate the existence of new health problems, and to guide the countermeasures of adverse reactions, medication management, and diet education; it also includes guidance on nutrition, exercise, and catheter maintenance. In the second week, the telephone return visit was conducted to evaluate the improvement of nursing problems existing in the first week of the return visit, mainly to strengthen the patients' health awareness, pressure for management, and timely dredge the patients' bad mood. Encourage patients to communicate with others and participate in normal social activities; guide patients to establish long-term life goals, and improve their recognition of their own value. Give psychological counseling to patients in bad mood and guide them to see a doctor if necessary. If the negative emotion of the patient is found in the intervention, which cannot be solved by simple telephone follow-up, it is necessary to conduct a targeted home visit. Family visits to all patients are completed by the researchers themselves. The specific time is one week after the second cycle of chemotherapy. Specific guidance is given in accordance with the patient's specific condition, the records of telephone return visits, and weekly questions. Make an appointment for a visit by phone first, and get to know the patient's problem by chatting and asking. The contents of the visit include assessment of patients' current and possible nursing problems, targeted provision of symptom-related knowledge, information and theoretical support, and corresponding guidance. The visiting time should not be too long, so as not to cause fatigue of the patients

### 2.3. Observation and Evaluation Indicators

#### 2.3.1. Satisfaction

After consulting the literature and experts' discussion, we designed patients' follow-up satisfaction, a total of 10 items, and recorded patients' satisfaction with follow-up management mode, health education, medical and nursing service, appointment registration process, and so on. It is divided into four dimensions: very satisfied, satisfied, general, and dissatisfied.

#### 2.3.2. Self-Management Efficacy Scale

The self-management efficacy of patients was evaluated on the day of admission, 1 day before discharge, as well as 1, 3, and 6 months after discharge. The Chinese version of Strategies Used by People to Promote Health [6] (SUPPH), contains 3 dimensions (self-decompression, positive attitude, and self-decision-making), with a total of 28 items, using a 5-grade score, including “lack of confidence” score 1 point, “have a little confidence” mean 2 points, “confident” mean 3 points, “very confident” scored 4 points, and “very confident” mean 5 points. The higher the total score, the higher the level of self-efficacy. ≤65 indicates low self-efficacy, 66-102 indicates moderate self-efficacy, and ≥103 indicates high self-efficacy. The Cronbach's *α* coefficient of the total scale was 0.970.

#### 2.3.3. Life Quality Scale of Lung Cancer Patients

The quality of life of the patients was evaluated on the day of admission, 1 day before discharge, as well as 1, 3, and 6 months after discharge. The Chinese version of the life quality scale for lung cancer patients [7] (QLQ-LC43) was employed to measure the life quality. QLQ-LC43 was divided into two parts: cancer patient quality of life scale (QLQ-C30) and lung cancer-specific model (QLQ-LC13). The life quality nuclear scale contains 30 items and 15 areas, including 5 functional areas, namely, patient physical function (PF), patient role function (RP), patient cognitive function (CT), patient emotional function (EF), and patient social function (SF), and 3 symptomatic areas, namely, patient fatigue (FA), patient pain (PA), and patient evil vomiting (NV). Six individual measurement items include insomnia (SL), dyspnea (DY), patient loss of appetite (AP), patient constipation (CO), patient diarrhea (DI), and patient financial difficulties (FI), each as a field, and an overall quality of life (QL) area. Functional areas include items 29-30 which are divided into 7 grades, 1-7 points, 1 for poor, 7 for good, and 4 for other items: never, a little, more, and a lot. The score is 1 to 4 directly. The higher the score, the better the quality of life.

#### 2.3.4. Mental Health

*(1)Anxiety*. The anxiety degree of the patients was accessed by the anxiety subscale of Hospital Anxiety and Depression Scale (HADS) [8] on the day of admission, 1 day before discharge, and 1 month after discharge. HADS is a short questionnaire consisting of 14 items, which has been widely used in clinic as a method to evaluate the bad mood of tumor patients. The anxiety subscale adopts a 4-grade scoring method, and the score range of each item is 0-3. The higher the score, the more serious the anxiety.

*(2)Depression*. On the day of admission, 1 day before discharge, and 1 month after discharge, the depression level of patients was measured by HADS depression subscale [9]. The depression subscale uses a 4-grade scoring system, and the score range of each item is 0-3. The higher the score, the more serious the depression. The average correlation coefficient of the two subscales of HADS was 0.56, and the coefficients of Cronbach's were 0.83and 0.82, respectively, which showed good reliability and validity.

#### 2.3.5. Family Care Index

The family care index [10] of the patients was evaluated on the date of admission, 1 day before discharge, and 1, 3 and 6 months after discharge. The family care index questionnaire is the questionnaire used to evaluate family function, including family fitness, cooperation, length, emotion, and intimacy, a total of 5 items; each item has 3 alternative answers: using the Likert 3 score method, select “often” to get 2 points, “sometimes” to get 1, and “never” to get 0. 0-3 was classified as severe, 4-6 as moderate, and 7-10 as good. The Cronbach's *α* coefficient of the scale is 0.78. It has good reliability and validity.

#### 2.3.6. Self-Transcendence Scale

Self-transcendence was evaluated on the day of admission, 1 day before discharge, and 1, 3, and 6 months after discharge. The self-transcendence scale [11] includes 15 items and adopted Likert 4-grade score: did not conform to the score of 1, only some conformed to 2 points, some conformed to 3 points, and very conformed to 4 points. The total score was 15-60 points. The higher the score, the higher the level of individual self-transcendence.

### 2.4. Statistical Analysis

The collected data were processed by SPSS24.0 software, and the counting data were presented by means of frequency and percentage; the measurement data were presented by mean ± SD; for the data in accordance with the normal distribution, *t*-test or *F*-test is adopted to test the statistics according to the different comparison groups; when *P* < 0.05, the difference was considered to be statistically significant.

## 3. Results

### 3.1. Comparison of Nursing Satisfaction

First of all, we surveyed the nursing satisfaction: of the study group, 24 cases were very satisfied, 5 cases were satisfied, and 1 case was general, and the satisfaction rate was 100%; of the control, 14 cases were very satisfied, 8 cases were satisfied, 4 cases were general, and 4 cases were dissatisfied, and the satisfaction rate was 86.67%. The nursing satisfaction of the study group was higher compared to the control, with significant difference (*P* < 0.05). All the data are illustrated in Figure 1.

### 3.2. Comparison of Self-Management Efficacy

Secondly, we compared the sense of self-management efficacy. On the day of admission, there was no evidently significant difference (*P* > 0.05). The scores of self-management efficacy at discharge and 1 month, 3 months, and 6 months after discharge were higher in the study group (*P* < 0.05). All the data are illustrated in Table 1.

### 3.3. Comparison of Quality of Life in Patients with Lung Cancer

Moreover, we compared the scores of quality of life, with no significant difference on the day of admission (*P* > 0.05). After nursing, compared to the control, the scores of quality of life of the two groups increased, and the scores of quality of life at discharge and 1, 3, and 6 months after discharge were greater of the study group (*P* < 0.05). All the data are illustrated in Table 2.

### 3.4. Mental Health Comparison

Next, we compared the mental health of the two groups, on the day of admission, with no significant difference (*P* > 0.05). Compared to the control, the anxiety and depression scores at discharge and 1, 3, and 6 months after discharge were lower of the study group (*P* < 0.05). All the data are illustrated in Table 3.

### 3.5. Comparison of Family Care Index

Next, we compared the family care index, on the day of admission, with no significant difference (*P* > 0.05). Compared to the control, the family care index at discharge and 1, 3 and 6 months after discharge was higher in the study group (*P* < 0.05). All the data are illustrated in Table 4.

### 3.6. Comparison of Self-Transcendence Scale

Finally, we compared the scores of the self-transcendence scale between the two groups, with no significant difference on the day of admission (*P* > 0.05). The scores of self-transcendence scale at discharge and 1, 3, and 6 months after discharge were greater in the study group compared to control (*P* < 0.05). All the data are illustrated in Table 5.

## 4. Discussion

Lung cancer ranks the most common lung malignant tumor, according to histological characteristics, which can be divided into small cell lung cancer (SCLC) and non-small cell lung cancer (NSCLC). About 80% of patients with lung cancer belong to NSCLC [12]. Due to the continuous deterioration of the global environment and the influence of poor lifestyle, the prevalence and mortality in lung cancer are elevating in recent years, ranking first in the malignancy related death; at present, lung cancer is considered to be the leading cause of cancer-related death in China [13]. Up to now, there were 733000 newly diagnosed patients with lung cancer in China in 2015, and 610000 people died of lung cancer [14]. Among female patients, the incidence of lung cancer ranks second among all malignant tumors, while the mortality rate ranks first. The life quality of patients with late lung cancer after chemotherapy has become the focus of public attention. Continuous nursing can provide patients with disease treatment, rehabilitation, and other useful information; meet their symptom management skills needs; ensure that patients get timely and continuous medical guidance; and improve their health outcomes. Therefore, the implementation of continuous nursing has become a general trend. At present, a number of scholars have carried out intervention studies on lung cancer patients undergoing chemotherapy in hospital, and the research on continuous nursing of lung cancer patients after discharge is relatively rare. Of note, the research on the application of perfect continuous nursing model to intervene patients with intermittent lung cancer chemotherapy is even more lacking [15, 16].

With the development of rehabilitation medicine, respiratory function training has been proposed as a way of lung rehabilitation training for patients undergoing lung cancer surgery, whose purpose is to enhance the strength and endurance of respiratory muscles through active breathing exercise, in order to lower the incidence of postoperative pulmonary complications and speed up the rehabilitation [17]. However, at present, there is no unified respiratory training standard or program for patients undergoing lung cancer surgery, and some commonly used methods include deep breathing training, balloon blowing, and breathing training apparatus. Compared with balloon blowing and breathing training, yoga breathing training does not require a specific device and is cost-effective. Meanwhile, compared with deep breathing training, yoga breathing training focuses not only on respiratory mechanics, but also on controlling every stage of breathing, and the use of breath timing in seconds is very important. This allows participants to inhale, hold their breath, and exhale in the best way during each breathing exercise. In addition, each breathing training method in yoga breathing training has specific effects [18]. For example, the complete breathing method in yoga breathing method can fully open the chest cavity through the combination of chest breathing method and abdominal breathing method, so that the main respiratory muscles of the human body, namely, diaphragm, intercostal muscle, and abdominal muscle, are involved in breathing exercise, so that the alveoli of the upper, middle, and lower lungs are involved in gas exchange, which can reduce dead space-like ventilation, improving ventilation and perfusion of poor pulmonary ventilation [18]. Clean breathing is a rapid abdominal breathing, through rapid abdominal contraction, pushing the diaphragm to squeeze the lungs so that respiratory secretions are excreted from the airway along with the air, which can reduce the retention of respiratory secretions; alternative nostril breathing alternately through the left and right nostrils for chest breathing can selectively activate the autonomic nervous system, resulting in a significant sedative effect [19]. However, patients' compliance with yoga breathing training is an important prerequisite to affect its effect. Some researchers have reported that patients' compliance with postoperative rehabilitation training is poor, and some reasons affecting compliance include the traditional belief that patients should stay in bed after surgery, and traditional health education is mainly based on individual knowledge indoctrination which cannot change the attitude and behavior of patients [20]. In addition, some patients can understand the importance of rehabilitation training, but they will encounter some problems that will reduce compliance during the training process, such as fear of wound pain, physical fatigue, depression, lack of supervision by medical staff, and lack of social support. Therefore, how to solve the problems encountered by patients in yoga breathing training more reasonably so as to improve patients' compliance with yoga breathing training is the key point [20]. ADOPT model is a problem-solving model put forward by American scholars in 2006. It consists of five steps: A (Attitude): individual attitude and expectation; D (Definition): individual identification of current obstacles and objective understanding of the nature of the problem; O (Open mind): individual thinking about new and creative ways to solve problems; P (Planning): individual determines feasible strategies; and T (Try it out). ADOPT model is incorporated into yoga breathing training for patients undergoing lung cancer surgery, in order to solve the problems encountered in yoga breathing training in time, make patients actively participate in breathing training and promote their rehabilitation [21].

Continuous nursing is through the development of a series of activity plans to ensure that patients receive continuous and collaborative care after discharge, which usually refers to the continuation of nursing from the hospital to the family [22]. The main purpose of continuous nursing is to carry out procedural education and guidance, so that patients can effectively solve their health problems after returning home from hospital, improve their self-care ability, promote the recovery of their physical function, and improve their quality of life [22]. Continuous nursing embodies the concept of patient-centered service; pays attention to the solution of health problems of discharged patients; aims to provide continuous, efficient, and comprehensive services for patients; and is the continuation and embodiment of high-quality nursing [22]. In 1947, the concept of continuous nursing was put forward for the first time in a report released by the American Joint Committee on Nursing Society and Health. The report points out that when patients are transferred from hospitals to families and communities, their treatment and care should not end and should be transferred with them, and nurses have an important role to play in the process; there is a need to provide continuous care guidance to patients [23]. In 1989, Pennsylvania College of Nursing carried out a landmark practice for the first time. Due to the continuous nursing service among discharged elderly patients, the readmission rate and disease recurrence rate of elderly patients were reduced. Therefore, this model has been valued and developed in many countries and regions. Continuous nursing, also known as extended nursing, is a nursing model that expands the scope of in-patient nursing services to families or communities. The more accepted definition can be traced back to 2003, and the American Geriatric Society defines it as a series of activities designed to provide continuous and coordinated care for patients when patients are transferred between different regions or between different health institutions. This continuity is mainly reflected in three aspects, including (1) the continuation of information, which means that caregivers can continuously get the patient's condition and health-related information, so as to provide patients with appropriate interventions; (2) the continuation of management, which continues to track changes in patients' physical conditions and care needs, as a basis for adjusting intervention strategies; and (3) the continuation of the relationship which means that a long-term therapeutic relationship is formed between the patient and the caregiver because of responsibility and trust [24, 25].

In terms of the results of our current study, nursing satisfaction in the study group was above that in the control. Our results indicated that the scores of self-management efficacy, quality of life, mental health, family care index, and self-transcendence scale in the study group were higher at discharge and 1, 3, and 6 months after discharge, compared to the control. Our results revealed that ADOPT nursing model plays a significant role in improving the quality of life of patients. Furthermore, our analysis shows that the respiratory training combined with continuous nursing based on ADOPT model constructed in this study is based on the concept of evidence-based and scientific and rigorous on the basis of consulting a large number of literatures. A multidisciplinary team has been set up, including doctors, nurses, counselors, and dietitians, to meet the health needs of patients. Before the implementation of the intervention, the members of the continuous intervention team completed standardized training to ensure the homogenization of the intervention. The whole process of intervention is led by competent nurses and oncology nurses with rich professional knowledge and clinical experience. Doctors provide professional support and dynamically adjust the intervention strategy according to the changes of patients' condition to ensure the correctness and effectiveness of the intervention. Through systematic evaluation and professional targeted guidance, patients can increase their knowledge of lung cancer disease and chemotherapy and improve their ability to deal with health problems, in order to facilitate their quality of life [26]. Our results indicated ADOPT mode combined with continuous nursing can improve the mental health and self-efficacy of lung cancer chemotherapy patients.

Taken together, patients with lung cancer chemotherapy using respiratory training based on ADOPT mode combined with continuous nursing can effectively facilitate the overall quality of life of lung cancer chemotherapy patients, can improve the mental health and self-efficacy of lung cancer chemotherapy patients, and then reduce the medical burden of patients. The nursing model based on ADOPT mode breathing training combined with continuous nursing is worth popularizing.

## Figures and Tables

**Figure 1:** Comparison of nursing satisfaction between two groups of patients.

**Table 1:** Comparison of self-management efficacy.

Group	*N*	Admission	Discharge	One month after discharge	3 months after discharge	6 months after discharge
Control	30	50.91 ± 3.11	55.96 ± 3.57	60.18 ± 4.23	65.87 ± 5.62	71.38 ± 4.12
Study	30	50.68 ± 3.51	60.81 ± 3.01	73.64 ± 3.67	86.84 ± 3.97	95.82 ± 4.97
*t*		0.268	5.688	13.164	16.692	20.735
*P*		0.789	<0.01	<0.01	<0.01	<0.01

**Table 2:** Comparison of quality of life in patients with lung cancer.

Group	*N*	Admission	Discharge	One month after discharge	3 months after discharge	6 months after discharge
Control	30	45.03 ± 4.36	50.98 ± 1.36	56.49 ± 3.56	60.84 ± 3.31	63.67 ± 3.16
Study	30	45.81 ± 4.31	56.73 ± 2.16	63.48 ± 3.16	70.73 ± 3.56	73.84 ± 3.45
*t*		0.696	12.338	8.042	11.143	11.906
*P*		0.488	<0.01	<0.01	<0.01	<0.01

**Table 3:** Comparison of quality of life scores in patients with lung cancer.

Group	*N*	Anxiety			Depression		
		Admission	Discharge	One month after discharge	Admission	Discharge	One month after discharge
Control	30	38.85 ± 2.54	35.91 ± 1.96	30.86 ± 3.19	40.87 ± 2.22	36.85 ± 2.67	35.28 ± 3.56
Study	30	38.98 ± 2.55	30.69 ± 3.51	26.97 ± 2.11	40.93 ± 2.33	32.69 ± 3.46	30.81 ± 2.11
*t*		0.197	7.111	5.570	0.012	5.213	5.916
*P*		0.843	<0.01	<0.01	0.919	<0.01	<0.01

**Table 4:** Comparison of family care index between the two groups.

Group	*N*	Admission	Discharge	One month after discharge	3 months after discharge	6 months after discharge
Control	30	4.06 ± 0.78	4.21 ± 0.46	4.68 ± 0.64	5.01 ± 0.17	5.18 ± 0.53
Study	30	4.09 ± 0.68	4.69 ± 0.67	5.19 ± 0.52	5.89 ± 0.77	6.58 ± 0.77
*t*		0.158	3.234	3.387	6.112	8.203
*P*		0.874	<0.01	<0.01	<0.01	<0.01

**Table 5:** Comparison of self-transcendence scale.

Group	*N*	Admission	Discharge	One month after discharge	3 months after discharge	6 months after discharge
Control	30	24.81 ± 4.91	30.84 ± 3.17	34.79 ± 3.17	37.49 ± 5.11	41.93 ± 3.17
Study	30	24.86 ± 4.18	36.94 ± 5.92	40.71 ± 5.92	45.83 ± 4.97	48.71 ± 2.94
*t*		0.042	4.975	4.828	6.408	8.589
*P*		0.966	<0.01	<0.01	<0.01	<0.01

## Data Availability

No data were used to support this study.
